The article "LncRNA NEAT1 enhances the radio-resistance of cervical cancer via miR-193b-3p/CCND1 axis" was retracted in 2023. Reasons: duplicated images; signs of a paper mill; unreliable data.

# LncRNA NEAT1 enhances the radio-resistance of cervical cancer via miR-193b-3p/CCND1 axis

**DOI:** 10.18632/oncotarget.23416

**Published:** 2017-12-18

**Authors:** Dongmei Han, Jianfeng Wang, Guanghui Cheng

**Affiliations:** ^1^ Department of Radiation Oncology, China-Japan Union Hospital of Jilin University, Changchun 130033, China

**Keywords:** lncRNA NEAT1, radio-resistance, cervical cancer, miR-193b-3p/CCND1 axis

## Abstract

LncRNAs have become a hot topic in various cancer-related researches. Radio-resistance is a great threat for cancer therapy. However, how lncRNAs affect the radio-resistance in cervical cancer is masked. As for our paper, it was discovered that NEAT1 was highly expressed in cervical cancer tissues and non-sensitive tissues as well as radio-resistant cell lines. And the overexpression of NEAT1 accelerated proliferation, while the knockdown of NEAT1 had the opposite result. The effect of NEAT1 on cell proliferation was dependent on the dose of ionizing radiation. And the silence of NEAT1 also caused cell cycle arrest in G0/G1 phase, and triggered more apoptosis, indicating the oncogenic role of NEAT1 in cervical cancer. Next, mechanistic assays affirmed that NEAT1 could function as a ceRNA to regulate cyclin D1 through sponging miR-193b-3p in cervical cancer. Rescue assays were employed to validate that miR-193b-3p and cyclin D1 could inhibit NEAT1-mediated suppressive effect on proliferation, and its stimulative effect on cell cycle arrest and apoptosis. In general, this article disclosed that NEAT1 could facilitate the radio-resistance of cervical cancer via competitively binding miR-193b-3p to up-regulate the expression of cyclin D1.

## INTRODUCTION

As one of the most familiar malignant cancers for the female, cervical cancer (CC) takes a great proportion of cancer-associated mortalities around the whole world [1, 2]. According to the survey, more than 529800 patients with cervical cancer are diagnosed every year and about 275100 of them face death [2]. Even though the patients suffering from cervical cancer can receive relevant treatments such as surgical operations, radiotherapy and chemotherapy, the positive survival fraction for them is still awful [1, 3]. Cervical cancer is still a big threat for women's health because of the limited medical technology. Therefore, a further study on the molecular mechanism of cervical cancer is urgently necessary.

Long non-coding RNAs are abbreviated as lncRNAs with a length more than 200 nt. LncRNAs have the ability to regulate gene expression in transcriptional and post-transcriptional levels via chromatin modification and genomic imprinting [4, 5]. There are varieties of researches reporting the relationship between lncRNAs and the carcinogenesis of many tumors, such as lncRNAs in breast cancer [6–8], lncRNAs in lung cancer [9], and lncRNAs in hepatocellular carcinoma [10]. Besides, there are also many papers discussing the functions of lncRNAs in cell cycle and differentiation [11] as well as in cell apoptosis [12, 13]. Thereby, it can be inferred that lncRNAs is a critical factor in dealing with the diseases associated with cancers. Here, we discussed the role of lncRNA NEAT1 in the radio-resistance of cervical cancer. It was discovered that NEAT1 was highly expressed in cancer tissues, non-sensitive tissues and radio-resistant cancer cells. NEAT1 enhanced the radio-resistance of cervical cancer through promoting cell proliferation, causing cell cycle arrest and triggering cell apoptosis.

MiRNAs, abbreviated from microRNAs, possess of about 20 nt. MiRNAs can activate or inhibit the 3’-UTR of downstream molecules in post-transcriptional level [14, 15]. And it has been demonstrated that miRNAs participate in the initiation and development of various cancers [16, 17], including cervical cancer [18, 19]. MiR-193b has been studied in multiple cancers including lung cancer [20], breast cancer [21], liposarcoma [22], and also cervical cancer [23, 24]. Despite there have been reports studying miR-193b in cervical cancer, the interaction of miR-193b with lncRNA NEAT1 in cervical cancer is unmasked. In this article, miR-193b-3p was negatively related to lncRNA NEAT1 and was able to directly spong with NEAT1 to activate the expression of its target gene in cervical cancer.

It has been demonstrated that miRNAs can participate in various cellular biological processes through sponging with 3’-UTR (3’-untranslated region) of target mRNAs, thus inducing the translational inhibition or degradation of mRNAs [25–28]. MRNA cyclin D1 (CCND1) is a vital promoter in the first central part of the Chr11q13 amplicon. And it has been decided that the abnormality of CCND1 is correlated to a range of human malignancies including lung cancer [29]. Nevertheless, the detailed information about the relationship between miR-193b-3p and CCND1 in cervical cancer is unclear.

As far as our study was concerned, we explored the roles of NEAT1, miR-193b-3p and CCND1 in cervical cancer independently. And we figured out that there existed a positive correlation between NEAT1 and CCND1, and a passive correlation between NEAT1 and miR-193b-3p. Furthermore, lncRNA NEAT1 could promote the radio-resistance of cervical cancer through competitively sponging with miR-193b-3p to regulate the expression of CCND1.

## RESULTS

### NEAT1 is elevated in cervical cancer tissues, non-sensitive tissues and radio-resistant cells

For a better understanding about whether lncRNA NEAT1 was involved in the radio-resistance of CC, we tested the expression level of NEAT1 in CC tissues and paired healthy tissues by means of qRT-PCR. It was clear that the level of NEAT1 in CC tissues was prominently higher than that in the healthy tissues (Figure 1A). On the basis of RECIST (Radiologic Response Evaluation Criteria in Solid Tumors), 72 pairs of cervical cancer tissues were classified into two groups, that is, radio-sensitive group and radio-non-sensitive group. It was observed that NEAT1 in the non-sensitive group was obviously more highly expressed than in sensitive group (Figure 1B). In addition, we also measured the expression of NEAT1 in the radio-resistant CC cell lines (HeLa (R) and SiHa (R)) and the matched parental cell lines (HeLa and SiHa). The expression level of NEAT1 was increased in the radio-resistant CC cells compared to that in the parental cells. All data in Figure 1 suggested that NEAT1 possibly participated in the radio-resistance of cervical cancer.

**Figure 1:** NEAT1 is elevated in cervical cancer tissues, non-sensitive tissues and radio-resistant cells **(A)** qRT-PCR was used to measure the expression level of NEAT1 in cervical cancer tissues and matched normal tissues. **(B)** qRT-PCR was used to measure the level of NEAT1 in sensitive and non-sensitive cancer tissues. **(C-D)** qRT-PCR was used to measure the level of NEAT1 in the radio-resistant cancer cells and their parental cells. All data were shown as mean ± S.D. from three independent assays. p<0.05^*^ and p<0.0.1^**^ were considered to be statistically significant.

### High level of NEAT1 marks the awful prognosis and responses to the radio-therapy

Kaplan-Meier curve analysis was applied to explore whether the survival rate of patients with CC was associated with the expression of NEAT1. As shown in Figure 2, patients with up-regulated NEAT1 had a poorer prognosis than those with down-regulated NEAT1 (P<0.001). Later, the relationship between NEAT1 expression and the clinical characteristics was analyzed. The mean value of NEAT1 expression was set as the threshold value, and the tissue specimens were divided into highly-expressed group (n=36) and under-expressed group (n=36). It was found that poor differentiation (p=0.003), TNM stage (p=0.001) and lymph node metastasis (p=0.002) rather than age, sex and smoking history (p>0.05) were associated with the high level of NEAT1 (Table 1). Besides, in accordance with RECIST, 59% of patients responded to radio-therapy completely or partially, while 41% of patients had no response to stable disease. Besides, NEAT1 closely related to therapeutic response was more up-regulated in non-responsive patients (p=0.016).

**Figure 2:** High level of NEAT1 marks the awful prognosis and responses to the radio-therapy Kaplan-Meier curve analysis demonstrated that patients with highly expressed NEAT1 had a poorer prognosis than those with under expressed NEAT1. Besides, poor differentiation, TNM stage, and lymph node metastasis were associated with the high level of NEAT1. And NEAT1 closely related to therapeutic response was more up-regulated in non-responsive patients.

**Table 1:** Correlation between lncRNA-NEAT1 expression and clinical features (n=72)

Variable	LncRNA-NEAT1 Expression		P-value
	low	high	
**Age**			
<60	17	14	0.634
≥60	19	22	
**Gender**			
Male	21	16	0.346
Female	15	20	
**Smoking**			
Smoking	14	19	0.344
No smoking	22	17	
**Differentiation**			
Well/Moderate	25	11	0.003^**^
Poor	11	25	
**TNM stage**			
I-II	25	10	0.001^**^
IIIa	11	26	
**Lymph metastasis**			
Absent	27	13	0.002^**^
Present	9	23	
**Treatment reponse**			
CR+PR	27	16	0.016^*^
SD+PD	9	20	

Low/high by the sample mean. Pearson χ^2^ test. P<0.05 was considered statistically significant.

### Enhanced NEAT1 strengthens the radio-resistance in cervical cancer cells

To investigate the effect of NEAT1 on the radio-resistance of CC, we transfected the radio-resistant cell lines (HeLa (R) and SiHa (R)) and their corresponding parental cell lines (HeLa and SiHa) with pcDNA-NEAT1 and specific si-RNA for NEAT1 (si-NEAT1#1, si-NEAT1#2) independently; in the meantime, the empty vector and control siRNA were used as negative controls. At 48 h after the transfection, the perfect transfection efficiency was obtained (Figure 3A). Subsequently, we explored how the transfection of NEAT1 influenced the biological behaviors in CC. Therefore, we employed MTT assay to determine the effect of NEAT1 on the sensitivity of CC cells to radiation. HeLa and SiHa cells were transfected with pcDNA-NEAT1 and then were exposed to different doses of ionizing radiation, exerting a dose-dependent suppressive effect on the cell proliferation. But the forced expression of NEAT1 reversed the suppressive effect slightly. On the contrary, HeLa (R) and SiHa (R) cells were transfected with si-RNAs and then were treated with different doses of ionizing radiation. However, compared to the negative control, the proliferation of the two radio-resistant cells transfected with si-NEAT1 were weak and were gradually attenuated with the increasing of the dose of ionizing radiation (Figure 3B). Soon after, we performed colony formation experiment to examine the effect of NEAT1 on the proliferation of CC cells treated with 2Gy of ionizing radiation. We discovered that the number of proliferative cells after the transfection with pcDNA-NEAT1 was much more than that in the negative control, which was inverse for the cells interfered with si-NEAT1 (Figure 3C).

**Figure 3:** Enhanced NEAT1 strengthens the radio-resistance in cervical cancer cells **(A)** HeLa and SiHa cells as well as HeLa (R) and SiHa (R) cells were transfected with pcDNA-NEAT1 and si-NEAT1 (si-NEAT1#1, si-NEAT1#2), with the empty vector or control siRNA as negative controls. **(B)** MTT assays were employed to examine the effect of NEAT1 on the sensitivity of cervical cancer cells to radiation. **(C)** Colony-formation assays were applied to test the effect of NEAT1 on cell proliferation treated with 2Gy of X-ray. All data were shown as mean ± S.D. from three independent assays. p<0.05^*^ and p<0.0.1^**^ were considered to be statistically significant.

### Silenced NEAT1 accelerates cell cycle arrest and triggers cell apoptosis

In order to make clear how NEAT1 touched off the radio-resistance in CC cells, we applied flow cytometry to analyze the cell cycle and apoptosis in CC. Remarkably, the down-regulation of NEAT1 increased the number of CC cells in G0/G1 phase and decreased the number of cells in S phase (Figure 4A). In conformity with the cell cycle analysis, western blot assay demonstrated a drooped protein level of the cyclin-dependent kinase (CDK2) and an improved level of p21 (Figure 4B). Next, apoptosis analysis revealed that the depressed NEAT1 induced much more apoptosis in radio-resistant CC cells (Figure 4C). Moreover, the protein levels of cleaved caspase-3 and caspase-9, two protein biomarkers for apoptosis, were lifted dramatically after the interference of si-NEAT1 (Figure 4D). These results testified that NEAT1 heightened the radio-resistance of CC cells through affecting cell cycle and apoptosis.

**Figure 4:** Silenced NEAT1 accelerates cell cycle arrest and triggers cell apoptosis **(A-C)** Flow cytometry was used to analyze the effect of NEAT1 on cell cycle (A) and cell apoptosis (C). **(B-D)** Western blot was performed to determine whether si-NEAT1 influenced the protein levels of CDK2 and p21 (B) as well as that of cleaved caspase-3 and cleaved caspase-9 (D). All data were shown as mean ± S.D. from three independent assays. p<0.05^*^ and p<0.0.1^**^ were considered to be statistically significant.

### NEAT1 directly binds to miR-193b-3p and is reversely related to miR-193b-3p

It had been reported that miR-193b could participate in the tumorigenesis together with lncRNAs in a ceRNA pattern [20]. Thus, it was hypothesized that there existed a cooperation between NEAT1 and miR-193b-3p. On the basis of the bioinformatics software (starBase), we obtained the predicted binging site (Figure 5A). Next, we designed the luciferase reporter analysis and RNA immunoprecipitation (RIP) assay to affirm our hypothesis. For the luciferase reporter analysis, the binding sites with the complementary sequence were cloned into the wild-type pmirGLO-NEAT1 vector (pmirGLO-NEAT1-WT), while the binding sites with the non-complementary sequence were constructed into the mutant-type pmirGLO-NEAT1 vector (pmirGLO-NEAT1-MUT). As illustrated in Figure 5B, miR-193b-3p mimics obviously weakened the luciferase activity of pmirGLO-NEAT1-WT rather than that of pmirGLO-NEAT1-MUT in HeLa (R) and SiHa (R) cells. In addition, the RIP assay showed that the fold changes of NEAT1 and miR-193b-3p in HeLa (R) and SiHa (R) cells were dramatically enriched in the beads containing Ago2 (Figure 5C). Then, we detected the expression level of miR-193b-3p in the parental cells (HeLa and SiHa) transfected with pcDNA-NEAT1, and that in HeLa (R) and SiHa (R) cells transfected with si-NEAT1. It was revealed that the overexpression of NEAT1 impaired the level of miR-193b-3p, whereas the knockdown of NEAT1 reinforced the level of miR-193b-3p, compared to those in the negative controls (Figure 5D). Such findings elucidated that NEAT1 suppressed miR-193b-3p to promote the radio-resistance in cervical cancer cells, proved by the result in the Spearman's correlation analysis (Figure 5E).

**Figure 5:** NEAT1 directly binds to miR-193b-3p and is reversely related to miR-193b-3p **(A)** The binding sites between NEAT1 and miR-193b-3p was obtained from the bioinformatics software (miRandSites). **(B-C)** Luciferase reporter analysis and RIP assay were applied to confirm the binding of NEAT1 to miR-193b-3p. **(D)** qRT-PCR was performed to measure the effect of NEAT1 on miR-193b-3p in cells transfected with pcDNA-NEAT1 and si-NEAT1. **(E)** Pearson's correlation analysis was performed to determine the relationship between NEAT1 and miR-193b-3p. All data were shown as mean ± S.D. from three independent assays. p<0.05^*^ and p<0.0.1^**^ were considered to be statistically significant.

### NEAT1 competitively sponges miR-193b-3p to enhance CCND1 in cervical cancer

It had been proved that NEAT1 could directly bind to miR-193b-3p to inhibit the suppressive function of miR-193b-3p in CC. In addition, it was found that CCND1 was one of the targets of miR-193b-3p by means of the bioinformatics software (miRandSites). And the potential binding sites between miR-193b-3p and CCND1 were shown in Figure 6A. Likewise, we also designed the luciferase reporter analysis to determine the relationship among miR-193b-3p, CCND1 and NEAT1. The plasmids including the complementary sequence were cloned into the wild-type pmirGLO-CCND1 vector (pmirGLO-WT-CCND1), while that including non-complementary sequence was cloned into the mutant-type pmirGLO-CCND1 vector (pmirGLO-MUT-CCND1). Consequently, miR-193b-3p mimics obviously lessened the luciferase activity of pmirGLO-CCND1-WT, which then was recovered by the overexpression of NEAT1. However, there were no obvious changes in the luciferase activity of pmirGLO-CCND1-MUT even with the overexpression of NEAT1 (Figure 6B). Soon after, we arranged the western blot assay to examine the protein level of CCND1 in HeLa (R) and SiHa (R) cells transfected with miR-193b-3p mimics and miR-193b-3p mimics plus pcDNA-NEAT1. It was clear that the reinforced expression of miR-193b-3p impaired the protein level of CCND1 in the radio-resistant cancer cells, which then was rescued a bit by pcDNA-NEAT1 (Figure 6C). These findings demonstrated that NEAT1 could enhance the expression level of CCND1 via acting as a ceRNA to sponge miR-193b-3p in CC.

**Figure 6:** NEAT1 competitively sponges miR-193b-3p to enhance CCND1 in cervical cancer **(A)** The binding site between CCND1 and miR-193b-3p was obtained from the bioinformatics software (starBase). **(B-C)** Luciferase reporter analysis and western blot assays were applied to confirm the relationship among NEAT1, CCND1 and miR-193b-3p. All data were shown as mean ± S.D. from three independent assays. p<0.05^*^ and p<0.0.1^**^ were considered to be statistically significant.

### Up-regulated CCND1 consolidates the radio-resistance of cervical cancer via influencing proliferation, cell cycle arrest and apoptosis

The expression level of CCND1 in CC tissues and cells was measured by qRT-PCR. CCND1 was up-regulated in CC tissues and cells (Figure 7A-7B). Then the effect of CCND1 on radio-resistant cancer cells was examined by means of MTT and colony formation assays for proliferation, and flow cytometry analysis for cell cycle and apoptosis. HeLa (R) and SiHa (R) cells were transfected with si-CCND1 and then were exposed to different doses of ionizing radiation. si-CCND1 transfection gradually decreased the survival fraction with the increase of the ionizing radiation (Figure 7C). Additionally, the knockdown of CCND1 also impaired the proliferative ability of HeLa (R) and SiHa (R) cells (Figure 7D). Furthermore, the decline of CCND1 resulted in the cell cycle arrest in G0/G1 phase, and caused more apoptosis (Figure 7E-7F). Based on these data, we presumed that CCND1 contributed to the NEAT1-mediated radio-resistance in CC. And the data from Spearman's correlation analysis ensured the positive correlation between NEAT1 and CCND1 (Figure 7G).

**Figure 7:** Up-regulated CCND1 consolidates the radio-resistance of cervical cancer via influencing proliferation, cell cycle arrest and apoptosis **(A-B)** CCND1 was up-regulated in CC tissues and cells, based on qRT-PCR. **(C-D)** si-CCND1 transfection gradually decreased the survival fraction with the increase of the ionizing radiation (C) and impaired the proliferative ability (D). **(E-F)** The decline of CCND1 resulted in the cell cycle arrest in G0/G1 phase, and caused more apoptosis. **(G)** Spearman's correlation analysis ensured the positive correlation between NEAT1 and CCND1.

### NEAT1 improves CCND1 to intensify the radio-resistance of cervical cancer through competitively sponging miR-193b-3p

To make certain the regulatory mechanism of NEAT1 in affecting the radio-resistance of CC, we arranged rescue assays in one CC cell (HeLa (R)). According to the MTT assay, with the increasing of the dose of ionizing radiation, the survival fraction in HeLa (R) cell transfected with si-NEAT1 became lower and lower compared to that in the negative control. But the gradually descended survival rate was saved somewhat by the inhibition of miR-193b-3p and the up-regulation of CCND1 (Figure 8A). Furthermore, as far as the colony formation assay was concerned, silenced NEAT1 decreased the number of the cloned cells compared with the negative control. However, the suppression of miR-139b-3p and the overexpression of CCND1 cancelled such an effect in HeLa (R) cell (Figure 8B). Next, it could be observed that the knockdown of NEAT1 induced cell cycle arrest in G0/G1 phase compared to that in the negative control, which was abolished by the repression of miR-139b-3p and the up-regulation of CCND1 (Figure 8C). And the apoptotic cells in HeLa (R) cell transfected with si-NEAT1 were much more than that in negative control; similarly, the increased apoptotic rate was abrogated by the descended miR-193b-3p and the strengthened CCND1 in HeLa (R) cell (Figure 8D). All of the data pointed out that lncRNA NEAT1 intensified the radio-resistance of CC through competitively sponging miR-193b-3p to improve the expression of CCND1.

**Figure 8:** NEAT1 improves CCND1 to intensify the radio-resistance of cervical cancer through competitively sponging miR-193b-3p **(A-D)** Rescue assays including MTT (A), colony formation (B), cell cycle (C) and cell apoptosis (D) were utilized to analyze the effect of the overexpression of CCND1 and the inhibitor for miR-193b-3p on the proliferation, cell cycle distribution and apoptosis rate in radio-resistant cells transfected with si-NEAT1. All data were shown as mean ± S.D. from three independent assays. p<0.05^*^ and p<0.0.1^**^ were considered to be statistically significant.

### Silenced NEAT1 impairs radio-resistance in cervical cancer *in vivo*

In order to figure out the effect of NEAT1 on the radio-resistance of CC cells *in vivo*, sh-NC cells and sh-NEAT1 cells were injected into the nude mice subcutaneously so as to obtain the xenograft mouse model. The efficient transfection was obtained by applying qRT-PCR (Figure 9A). Obviously, with the increasing of the radiation ionizing, both the tumor volume and weight were decreased; furthermore, the knockdown of NEAT1 made volume and weight smaller and lighter (Figure 9B-9C). In addition, the expressions of miR-193b-3p and CCND1 were examined after the silence of NEAT1 *in vivo*. As illustrated in Figure 9D, silenced NEAT1 enhanced the expression of miR-193b-3p but attenuated the expression of CCND1 *in vivo*, compared to the negative controls. Such data explained that NEAT1 promoted the radio-resistance of CC cells *in vivo* through suppressing miR-193b-3p to up-regulate the expression of CCND1.

**Figure 9:** Silenced NEAT1 impairs radio-resistance in cervical cancer *in vivo* **(A)** The efficient transfection was obtained by applying qRT-PCR. **(B-C)** Both the tumor volume and weight were decreased; furthermore, the knockdown of NEAT1 made volume and weight smaller and lighter. **(D)** Silenced NEAT1 enhanced the expression of miR-193b-3p but attenuated the expression of CCND1 *in vivo*. All data were shown as mean ± S.D. from three independent assays. p<0.05^*^ and p<0.0.1^**^ were considered to be statistically significant.

## DISCUSSION

LncRNAs are famous for its ability to regulate the mRNA and protein levels of sundry target genes and their physiological processes [30, 31]. And it is also well-known that lncRNAs are responsible for the tumorigenesis of various tumors as oncogenes or tumor suppressors [32]. LncRNA NEAT1 has been studied to be an oncogene in numerous cancers such as breast cancer [33], non-small cell lung cancer [34], and hepatocellular carcinoma [35]. However, the detailed description about lncRNA NEAT1 in cervical cancer is not clear.

Additionally, a quantity of researchers have validated that miRNAs are outstanding in mediating the biological behaviors like the cell proliferation, migration and invasion and so on through interacting with their downstream targets in quantities of cancers [36, 37]. For example, miR-221/222 promotes the proliferation of breast cancer by regulating PTEN [38]; miR-155 represses the growth of lung cancer via targeting PDCD4 [39]; miR-1236-3p inhibits the metastasis and invasion of LAD cells by regulating KLF8 [40]. But how miR-193b-3p affects the progress of cervical cancer is not sure.

CCND1 is a critical protein in regulating cell cycle. And its dysregulation has been proved to be tied to different malignant cancers. For example, CCND1 cooperates with the EMSY gene in the carcinogenesis of non-small cell lung cancer [29]. But the role of CCND1 in cervical cancer is masked.

On behalf of two extremely vital non-coding RNAs, lncRNAs and miRNAs take charge of various processes of tumors, even in a cooperative manner with the downstream molecules of miRNAs. And it has been acknowledged that lncRNAs can function as ceRNAs through sponging with miRNAs to up-regulate multiple mRNAs. For example, Zhaoliang Chen et al. studied that lncRNA TINCR regulated PDK1 via acting as ceRNA to bind miR-375 in GC [41]; Li RK et al. reported that PTENP1 regulated PTEN through competitively binding miR-19b in BC [42, 43]. In speaking of lncRNA NEAT1, its function as a ceRNA in cervical cancer has not been discussed clearly.

As to this paper, we firstly measured the expression levels of NEAT1 in CC tissues, non-sensitive tissues and radio-resistant cells. It was found that NEAT1 was up-regulated in the above tissues and cell lines. And the overexpression of NEAT1 improved the survival rate in an ionizing radiation-dependent manner, while the silence of NEAT1 decreased the survival rate in the ionizing radiation-mediated way. Equally, we got the similar results from the same experiments for CCND1. It was also notarized that NEAT1 was positively associated with CCND1 but was negatively connected with miR-193b-3p. Besides, we confirmed that NEAT1 could regulate CCND1 by sponging miR-193b-3p in cervical cancer, ensured by the bioinformatics software, luciferase reporter analysis and RNA immunoprecipitation assay as well as a series of rescue assays. What's more important, all of the biological behaviors induced by lncRNA NEAT1 were relied on the doses of ionizing radiation. Moreover, it was also clarified *in vivo* assays that NEAT1 suppressed the level of miR-193b-3p to enhance the expression of CCND1 in CC cells. Thus, we concluded that lncRNA NEAT1 might act as a ceRNA to promote the radio-resistance of cervical cancer by competitively binding to miR-193b-3p to regulate the expression of CCND1.

## MATERIALS AND METHODS

### Patient's samples

Totally, we collected 72 pairs of brand-new CC tissue samples and matched normal tissue samples from patients having suffered from surgical operations in the Department of Radiation Oncology, China-Japan Union Hospital of Jilin University, Jilin, Changchun, China. All the samples were conserved at 80 degrees below zero. All the processes involved in the study were agreed by the Research Ethics Committee of China-Japan Union Hospital of Jilin University. Every patient was offered a written informed consent.

### Cell lines

Two human CC cell lines (HeLa and SiHa) were provided by American Type Culture Collection (ATCC, USA). The radio-resistant cells called after HeLa (R) and SiHa (R) sprang from the dose-gradient irradiation. HeLa and SiHa cells as well as HeLa (R) and SiHa (R) were treated in a RPMI 1640 medium (Invitrogen, USA) with 10% of fetal bovine serum (FBS; Gibco, USA), penicillin (100 U/mL), and streptomycin (100 μg/mL). All of the cells were saved in a humid air at 37°C with 5% of CO^2^.

### Cell transfection

In order to up-regulate NEAT1, we made the plasmid with the full-length coding sequence of NEAT1 to be cloned into the pcDNA 3.0 vector (Realgene, Shanghai, China) and the entirety was enlarged in accordance with the manufacturer's guidance. The siRNAs for NEAT1, CCND1 and scramble negative control as well as miR-193b-3p inhibitor were obtained from Invitrogen and transfected into cells by means of Lipofectamine 2000 (Invitrogen, Carlsbad, CA, USA) according to the manufacturer's requirements.

### Quantitative real-time reverse transcription PCR (qRT-PCR)

On the basis of the manufacturer's proctols, all RNAs were extracted by using the TRIzol reagent (Invitrogen, USA). 1 μg of total RNAs was inversely transcribed by means of random primers, with the help of the RevertAid First Strand cDNA Synthesis kit (Thermo Fisher Scientific, USA). According to the previous description [44], we took advantage of the SYBR-Green PCR Master Mix kit (Takara, Japan) to test the mRNA levels of miR-193b-3p and CCND1. The primers used in this experiment were as the listed: GAPDH (forward): 5’-CCTCGTCTCATAGACAAGATGGT-3’, (reverse): 5’-GGGTAGAGTCATACTGGAACATG-3’; NEAT1 (forward): 5’- TCGGGTATGCTGTTGTGAAA-3’, (reverse): 5’- CGTAACAGAATTAGTTCTTAC-3’; miR-193b-3p (forward): 5’- TCTACAGTGCACGTGTC TCCAG-3’, (reverse): 5’- ACCTGCGTAGGTAGTTTCA TGT-3’; CCND1 (forward): 5’- TCCTACTACCGCCTCA CA-3’, (reverse): 5’- ACCTCCTCCTCCTCCTCT-3’. All of the data were expressed as the mean ± SD for at least three independent experiments, and 2^−ΔΔCt^ method was used to measure the relative levels of genes.

### Proliferation assays

For MTT assay, cells sensitive to the radio-therapy were treated with 3-(4, 5-dimethylthiazol-2-yl)-2, 5-diphenyl-trtrazolium bromide. We sealed 5 × 10^3^ cells/well in a 96-well plate for 24 h, and then transfected them with ordered vectors and finally made them to be cultured in a normal medium. Next, cells after being transfected were exposed to different doses of ionizing radiation from 0 Gy to 10 Gy. And then each well in the plate was supplemented with MTT solution (5 mg/ml, 20 μl). 4 h later, we took away the medium and added 100 μl DMSO into each well. In the end, the optical density of cell lysates at 560 nm was used to measure the number of the survived cells. All experiments were carried out for at least three times.

For colony formation assay, we placed 500 cells per well into the 6-well plates and cultured them in a normal medium at 37°C. 2 weeks later, the cells were fixed and dyed with 0.1% of crystal violet. Finally, the visible cloned cells were counted manually.

### Flow cytometry analyses

For the cell apoptosis analysis, we made use of the Annexin V: FITC Apoptosis Detection Kits (BD Biosciences, USA), in the light of the manufacturer's instructions.

For cell cycle distribution analysis, we gathered transfected cells immediately after the transfection and washed them with ice-cold phosphate-buffered saline (PBS), and then fixed them with 70% of ethanol for a whole night at -20°C. Later, we rehydrated the fixed cells in PBS for 10 min which then were cultured in RNase A (1mg/ml) for 30 min at 37°C, followed by their subjection to PI/RNase staining. Finally, the cells were analyzed under the help of a FACScan instrument (Becton Dickinson, Mountain View, CA) and the Cell Quest software (Becton Dickinson, San Jose, CA).

### Western blot

HeLa and SiHa cells were lysed with a lysis buffer containing the protease inhibitor cocktail (Sigma-Aldrich, USA). The proteins with the same concentrations were split with 8% of SDS/PAGE gels, and then were transported to PVDF membranes (Millipore, USA). The PVDF membranes were incubated with the primary antibodies at 4°C for a whole night. The treated PVDF membranes were cultured with secondary antibodies that were conjugated with HRP for 1 h with the room temperature. Here were the necessary primary antibodies: anti-rabbit-p21 (1:1000 dilutions, Santa Cruz, USA), anti-rabbit-CDK2 (1:1000 dilutions, Cell Signaling Technology, Beverly, MA, USA), anti-rabbit-cleaved-caspased-3 antibody (1:1000 dilutions, Cell Signaling Technology, Beverly, MA, USA), anti-rabbit-cleaved-caspased9 antibody (1:1000 dilutions, Cell Signaling Technology, Beverly, MA, USA), and anti-rabbit-GAPDH antibody (1:5000 dilution, Cell Signaling Technology, Beverly, MA, USA).

### Luciferase reporter analyses

Luciferase reporter analyses were used to detect the binding among NEAT1, miR-193b-3p and CCND1. Therefore, we amplified the sequences including the predicted binding sites of miR-193b-3p for NEAT1-WT, NEAT1-MUT, CCND1-WT, and CCND1-MUT. Then the sequences were subcloned into the pmirGLO-control vectors (Promega, Madison, WI, USA). The reporter vectors with miR-193b-3p and miR-control were co-transfected into HeLa and SiHa cells by using Lipofectamine 2000 (Invitrogen). 36 h later, we gathered the lysed cells and detected the luciferase activity by means of the Dual-Luciferase Reporter Assay System (Promega).

### RAN immunoprecipitation (RIP) assay

For the RIP assay, we used the EZ-Magna RIP RNA-binding protein immunoprecipitation kit (Millipore, USA). Then, HeLa and SiHa cells were lysed by using RNA lysis buffer including the protease and RNase inhibitors. Different cell lysis solutions were cultured by means of the magnetic beads coated with anti-human argonaute 2 (Ago2) antibodies (Millipore, USA) for RIP buffer. IgG (Millipore, USA) was regarded as a negative control. In the end, after 2 h of incubation at 4°C, the co-precipitated RNAs were extracted and the unbound materials were removed, followed by the reverse transcription and PCR analysis.

### Xenograft in nude mice

Recombinant lentiviruses including sh-NC and sh-NEAT1 (5’- GCCATCAGCTTTGAATAAATT-3’) were provided by the GeneChem Company (Shanghai, China), followed by their transfection into radio-resistant CC cells. As to *in vivo* assays, 5-week-old male athymic nude mice (BALB/c nu/nu), kept under the specific-pathogen-free conditions with a light/dark cycle of 12/12 h, were offered with standard chow diet and water. 1×10^7^ sh-NC and sh-NEAT1 cells were injected subcutaneously into the mice treated with different doses of ionizing radiation. Tumor growth was examined by means of calipers with the increasing of ionizing radiation. After 32 days of transplantation, the mice were sacrificed to analyze the tumor weight. All animal assays were approved by the Institutional Animal Care and Use Committee of China-Japan Union Hospital of Jilin University.

### Statistical analysis

All of the data were presented as mean ± standard deviation. And all assays were performed for three times independently. The differences between the two groups were analyzed with the Student's t-test, while the differences among 3 or more groups were measured by using one-way analysis of variance with SPSS 19.0. P-value < 0.05 was considered statistically significant.
